The article "Recombinant production of eukaryotic cytochrome P450s in microbial cell factories" was published in 2018. Journal: Biosci Rep.

# Recombinant production of eukaryotic cytochrome P450s in microbial cell factories

**DOI:** 10.1042/BSR20171290

**Published:** 2018-03-05

**Authors:** Johanna Hausjell, Heidi Halbwirth, Oliver Spadiut

**Affiliations:** TU Wien, Institute of Chemical, Environmental and Biological Engineering, Vienna, Austria

**Keywords:** Cytochrome P450, Escherichia coli, Pichia pastoris, recombinant protein, Saccharomyces cerevisiae

## Abstract

Cytochrome P450s (P450s) comprise one of the largest known protein families. They occur in every kingdom of life and catalyze essential reactions, such as carbon source assimilation, synthesis of hormones and secondary metabolites, or degradation of xenobiotics. Due to their outstanding ability of specifically hydroxylating complex hydrocarbons, there is a great demand to use these enzymes for biocatalysis, including applications at an industrial scale. Thus, the recombinant production of these enzymes is intensively investigated. However, especially eukaryotic P450s are difficult to produce. Challenges are faced due to complex cofactor requirements and the availability of a redox-partner (cytochrome P450 reductase, CPR) can be a key element to get active P450s. Additionally, most eukaryotic P450s are membrane bound which complicates the recombinant production. This review describes current strategies for expression of P450s in the microbial cell factories *Escherichia coli, Saccharomyces cerevisiae*, and *Pichia pastoris*.

## Introduction

Cytochrome P450s are present in all kingdoms of life and make up one of the largest and most diverse known protein families. P450s contain an iron–porphyrin group incorporated in their core and are therefore classified as hemoproteins. Their name results from a characteristic absorption band, which they exhibit when complexed with carbon monoxide. Absorption of blue light at 450 nm destroys the enzyme—carbon monoxide complex and thereby restores catalytic activity [1].

P450s catalyze monooxygenase reactions, more particularly, the hydroxylation or epoxidation of hydrocarbons. Oxygen is activated by the enzymes to react with unactivated C–C and/or C–H bonds [2]. P450-catalyzed reactions are involved in many essential processes comprising carbon source assimilation, synthesis of hormones and secondary metabolites, carcinogenesis, and degradation of xenobiotics [1]. An exemplary reaction from steroidogenesis, catalyzed by CYP11B1 (steroid 11-β-hydroxylase), is shown in Figure 1.

**Figure 1:** Exemplary reaction catalyzed by a P450 11-desoxycorticosterone is hydroxylated at position 11 by CYP11B1 leading to corticosterone.

Due to the intrinsic ability of P450 enzymes to specifically hydroxylate complex hydrocarbons, attainment of high amounts of P450s is of interest in regard to biotransformations and industrial applications. Possible implementations include the production of drugs, vitamins, flavors, fragrances, and pesticides [3]. Isolation of P450s from native tissues, however, often only results in modest yields, therefore, recombinant protein production is an attractive alternative. Aside from employment of P450s as catalysts, another incentive for recombinant production is, in many cases, the elucidation of the protein structure and/or function. Therefore, the rather challenging and laborious approach of recombinant expression of soluble protein and subsequent crystallization has to be undertaken. In Figure 2, the crystal structure of yeast lanosterol 14α-demethylase, a member of the CYP51 family, which was crystallized including its N-terminal anchor, is shown.

The article "Recombinant production of eukaryotic cytochrome P450s in microbial cell factories" was published in 2018. Journal: Biosci Rep.

**Figure 2:** Exemplary crystal structure of a P450 Structure of lanosterol 14α-demethylase (PDB 4LXJ), a P450 crystallized including its membrane anchor (circled in red).

However, the attainment of sufficient quantities of active P450 enzymes, for either structure–function elucidation or industrial implementation, entails many challenges: factors impeding expression include the incorporation of the heme group, the requirement of a redoxpartner (cytochrome P450 reductase (CPR) for eukaryotic P450s), as well as the fact that most eukaryotic P450s are membrane bound [4,5]. Here, we present a review of strategies developed for the production of eukaryotic P450s in the microbial cell factories *Escherichia coli, Saccharomyces cerevisiae*, and *Pichia pastoris*. The different strategies are described and contrasted and the different expression hosts are evaluated. This review provides a compact overview of available strategies for the enhanced recombinant expression of active P450s in *E. coli, S. cerevisiae*, and *P. pastoris* and serves as a guideline for choosing expression strategies for the production of eukaryotic P450s in heterologous hosts.

## Strategies for P450 production in microbials

### E. coli

*E. coli* as expression host is often the first choice when recombinantly producing proteins. There are numerous established methods for genetic manipulation and the organism is fast growing on inexpensive media up to high cell densities [6–8]. All of this leads to high yields of recombinant protein. However, challenges are faced when expressing more complicated eukaryotic proteins in *E. coli*. The bacterium is not able to perform most post-translational modifications, and expression of membrane proteins is not trivial, as *E. coli* lacks the inner organelles in which eukaryotic membrane proteins are anchored [5]. An exemplary illustration of a eukaryotic cell with the anchoring of a membrane protein is shown in Figure 3.

The article "Recombinant production of eukaryotic cytochrome P450s in microbial cell factories" was published in 2018. Journal: Biosci Rep.

**Figure 3:** P450 location in a eukaryotic cell Schematic picture of a eukaryotic cell (left) and the anchoring of an exemplary membrane protein (right) with catalytic domain (red) and its membrane anchor (green).

In spite of being membrane proteins, numerous eukaryotic P450s have been successfully expressed in *E. coli* using different approaches as also reviewed by Zelasko [9]. An overview of the most frequently used strategies is given in Figure 4.

**Figure 4:** Strategies for recombinant expression of P450s in *E. coli* Overview of strategies applied for the expression of P450s in *E. coli.*

#### N-terminal modifications

Most eukaryotic P450s are membrane bound, the majority of them being natively located in the endoplasmic reticulum, whereas a few are found in the mitochondria of eukaryotes. The N-terminal region of those P450s comprises a transmembrane helix, responsible for anchoring [10]. This comparatively hydrophobic domain impedes production in *E. coli* considerably.

When expressing membrane bound proteins in *E. coli*, most often a high amount of insoluble protein aggregates, so called inclusion bodies, are formed. This is due to the fact that *E. coli* lacks inner organelles and thus the native protein cannot be properly incorporated into membranes. Consequently, the hydrophobic regions are displayed and agglomerate to inclusion bodies [5].

This obstacle is most frequently overcome by performing modifications at the N-terminus: either by altering the sequence in the 5′ region of the DNA or by removal of the membrane anchor.

##### N-terminal sequence change

When it comes to sequence exchanges at the N-terminus, the sequence that is by far the most often used is MALLLAVF(L): it originates from a bovine P450 (P450 17A), and has been proven effective for enhancing solubility in numerous cases [11–15]. The sequence was first introduced by Barnes et al. [16], who showed that only slight alteration of the 5′ DNA-sequence can allow integration of P450s into the outer membranes of *E. coli*. The production of 16 mg active P450 per liter of culture was achieved by mutating the sequence 5′ from ATGTGGCTGCTCCTGGCTGTCTTT to ATGGCTCTGTTATTAGCAGTTTTT or in terms of amino acids from MWLLLAVF to MALLLAVF.

Exchanging the N-terminus of other eukaryotic membrane bound P450s to this sequence has been proven effective in many cases: Pan et al. [11] used the sequence for successful expression of two human cytochromes (P450 2D6 and CYP3A4), which yielded around 20 mg/l culture in both cases. Cheesman et al. [13] achieved expression of 460 nmol/l of CYP6G1 stemming from *Drosophila melanogaster* when exchanging the N-terminus from MVLTEVLFF to MALLLAVF; however, they found the larger part of the protein to be located in the cytosolic fraction (122 nmol in membrane fraction vs 288 nmol in the cytosolic fraction). Hanna et al. [17] used the MALLLAVF sequence for expression of human P450 2B6; however, expression was only successful by further adding chloramphenicol to the media, which induced cold-shock proteins, and thus enhanced proper folding. Sandhu et al. [18] found several human P450s expressed at higher levels when exchanging the N-terminus to MALLAVF. Wang et al. [15] found the same for rat CYP3A9. Haudenschild et al. [14] tested various N-terminal modifications for limonene hydroxylase from mint, and also found the highest expression level when exchanging the N-terminal sequence to the MALLLAVF sequence. Similarly, Tang et al. [12] tried different N-terminal amino acid exchanges, and again found the construct with the bovine N-terminal sequence to be expressed at the highest level.

The article "Recombinant production of eukaryotic cytochrome P450s in microbial cell factories" was published in 2018. Journal: Biosci Rep.

Gillam and co-workers did more extensive research on N-terminal modifications of P450s: apart from exchanging the N-terminal sequence to the MALLLAVF sequence, they performed additional alterations further downstream of the 5′ sequence for P450 3A7 and P450 3A5 (both human P450s) and showed that this could further elevate hemoprotein yields [19,20]. For three other human P450s (P450 2D6, 3A4, and 2E1), they showed that deletions in the N-terminal region led to higher expression yields [21–23].

Ichinose et al. [24] performed large scale expression screenings of several hundred modified P450s for identification of potential chimeric partners for the heterologous expression of fungal P450s in *E. coli*. In 2013, they screened expression of 304 fungal P450 isoforms: they identified 23 that were expressible with simple deletions at the N-terminus and 4 that were expressible without N-terminal modifications. The latter exhibited N-terminal sequences that can be potentially used for construction of chimeric P450s, expressible in soluble form. In 2015, they extended their screening experiments and identified further 64 potential chimeric partners for expression in *E. coli*. They also showed that several fungal P450s could be expressed when their N-terminal domain was replaced by the one of CYP5144C1 [25]. In 2016, Hatakeyama et al. [26] showed that N-terminal sequence exchange led to a more than 6-fold increase in product yield for the fungal P450 CYP136A1 and allowed expression of CYP5136A3, which was not expressible without modifications.

Another strategy, namely fusing the N-terminus of the P450 to sequences of bacterial proteins, has been extensively studied by Vazquez-Albacete et al. [27], who used C-terminal GfP-fusions of plant cytochrome P450 CYP79A1 for analyzing expression levels. They created P450 fusions with bacterial membrane anchors with the C-terminus facing the cytoplasmic site, bacterial membrane proteins with the C-terminus facing the periplasmic site, bacterial signal peptides, and bacterial transporters. They found that, compared with the wild type, all fusions led to increased expression of P450. Most successful were the fusions to membrane anchors with the C-terminus facing the cytoplasmic site, especially the YcjF variant followed by fusions with signal peptides.

The article "Recombinant production of eukaryotic cytochrome P450s in microbial cell factories" was published in 2018. Journal: Biosci Rep.

##### N-terminal deletion

In many cases also N-terminal deletions have proven effective for successful expression of P450s in *E. coli*: Ahn et al. [28] showed the successful expression of human cytochrome P450 1A2 with an N-terminal truncation, which could be further enhanced (3.5-fold) by coexpression of chaperones. In the expression of CYP3A37, Rawal et al. [29] achieved to up to 250–400 nmol/l by deleting 11 amino acids in the N-terminal region, whereas the native version did not express at all. Park et al. [30] compared the expression of native P450 2J2 to one with a MALLLAVF sequence and one with a 34 amino acid deletion. They found that the native one could not be expressed, while the variant with the MALLLAVF sequence was expressed at 120 nmol/l of cell culture. However, the variant with the deletion in the N-terminus was even expressed at 320 nmol/l cell culture, while still exhibiting the same characteristics as the native protein.

However, it also has to be mentioned that N-terminal deletion can lead to loss of function in some cases, as for example shown by Doray [31].

#### Coexpression of auxiliary proteins

For the majority of P450s a redox-partner, CPR, is needed to catalyze the monooxygenase reactions [1]. Their interaction is schematically depicted in Figure 5.

**Figure 5:** Interaction of P450 and CPR Schematic representation of the interaction between P450s (red, PDB 4K9T) and CPRs (green, PDB 3QE2). The CPR reduces NAD(P)H and thereby provides the P450 with electrons for the oxidation of substrates.

The CPR provides the necessary equivalents of NADP, which is in turn reduced by the P450 when oxidizing the hydrocarbon [32]. When P450s are overexpressed, their need for NADP can stress the organism, and cause a metabolic imbalance. Therefore, a frequently used strategy is the co-overexpression of CPRs. In most cases, the reductase is co-overexpressed [11,12,26,29,33–39]. Less commonly, the P450 is expressed as a fusion protein together with the reductase [40,41].

The article "Recombinant production of eukaryotic cytochrome P450s in microbial cell factories" was published in 2018. Journal: Biosci Rep.

Aside from CPRs also the coexpression of chaperones, most frequently GrOES/EL [42] can lead to an increased yield of active protein.

##### Coexpression of CPR

Strategies for coexpression of CPRs include expression as a fusion protein, expression of both proteins from a bicistronic plasmid (where the P450 and its reductase are expressed from the same promoter which is followed by two ribosome-binding sites), expression of the proteins from one plasmid with two promoters, or expression from two independent plasmids [11]. Those techniques have often been used to either investigate the function of an unknown P450 or for whole cell catalysis: Crewe et al. [33] for instance expressed 12 different P450 enzymes, each from a bicistronic plasmid, together with recombinant human NADPH–cytochrome P450 reductase to find the ones involved in tamoxifen metabolism. Josephy et al. [43] simultaneously expressed CoA:arylamine N-acetyltransferase, human cytochrome P450 1A2, and NADPH–cytochrome P450 reductase to create a strain that is able to convert aromatic amines into reactive, mutagenic N-acetoxy esters. Lee et al. [44] used coexpression of P450 and reductase in order to characterize the Ala62Pro polymorphic variant of human cytochrome P450 1A1 and Palma [33] used it to characterize eight polymorphic forms of human CYP1A2.Quehl et al. [38] coexpressed human cytochrome P450 1A2 and cytochrome P450 reductase on the cell surface of *E. coli* to develop a system for investigation of drug metabolism. Hernandez-Martin et al. [45] even used a tricistronic plasmid, expressing CYP154E1, together with two redox partners (Pdx/Pdr and YkuN/FdR), for whole cell biotransformation of Grundmann’s ketone.

Fusions of reductase and hydroxylation domains have been employed by Leonard et al. [40] and Nodate et al. [41], who both fused the reductase domain to the P450 to be expressed.

However, it is also reported that coexpression of reductase and P450 leads to lower yields in P450 production [13], which might be explained by the additional burden on the organism of overexpressing a second recombinant protein.

##### Coexpression of other redox-partners and Cyt b5

Another interesting approach to compensate for the missing redox-partner when overexpressing P450s in *E. coli* was demonstrated by Lu et al. [46] where glucose dehydrogenase was coexpressed to provide the additional NADP molecules needed. Dong et al. [34] found coexpression with cytochrome *b*5 to increase product yields by 20–60%, as a result of mRNA stabilization.

##### Coexpression of chaperones

A frequently observed bottleneck when recombinantly expressing proteins in *E. coli* is the proper folding, as the native folding mechanism of *E. coli* cannot keep up with the speed of transcription and translation [47]. Hence, coexpression of chaperones often results in higher amounts of properly folded, and thus active, protein. Therefore, pGro plasmids are often employed when expressing complex proteins such as P450s to facilitate coexpression of the GroEL/GroES chaperones [13,24–26,48].

The article "Recombinant production of eukaryotic cytochrome P450s in microbial cell factories" was published in 2018. Journal: Biosci Rep.

#### Media supplementation with ALA

When actively producing P450s in *E. coli*, the incorporation of the heme group into the core of the enzyme is a major challenge. This is why a heme-precursor, δ-ala-leuvenic acid, is usually supplied to the media [13,24–26,28,45]. This precursor has in several cases been shown to be beneficial for increased expression of active P450s [49,50].

#### Cultivation parameter optimization

Another illegibly contributing factor in expression optimization is the adjustment of cultivation parameters [7] ranging from temperature, pH levels, to inducer and dissolved oxygen concentrations.

Faiq et al. [49] wanted to express native cytochrome P450 1B1 (without any N-terminal modifications) and therefore investigated different cultivation parameters, which are summarized in Table 1. Lu and Mei [46] similarly investigated expression parameters with the pET-based BL21(DE3) expression system. The parameters investigated, and their effects are also found in Table 1, with the optima in bold.

**Table 1:** Cultivation parameters compared for expression of P450, optimum-found shown in bold letters

Reference	Strains	Plasmids	Time (h)	IPTG-conc. (mM)	RPM (1/min)	Temperature (°C)	δ-ALA-conc. (mM)	Thiamin-conc. (mM)
[46]	BL21(DE3)	pET28a	2	0.2		25		
			4	**0.5**		**30**		
			6	0.8		34		
			**8**	1		37		
			10					
[49]	**JM109**	**pCWori**	12	0.2	150	18	0.2	0.5
	DH5α	pET28a	20	0.4	**170**	25	0.4	1
	C100	pTreHis	**24**	**0.6**	200	**30**	0.6	1.5
	DE3		30	0.8	250	37	**0.8**	
	CodonPlus							
	Pril							

Abbreviation: IPTG, isopropyl-β-D-thiogalactopyranoside

As shown in Table 1, similar IPTG-concentrations (0.5 and 0.6 mM) and the same temperature (30°C) were found to be optimal. However, it is hard to compare these parameters, as different expression systems have been used.

Several groups found the dO_2_ concentration to have an impact; however, the results are contradictory. Zhang and co-workers reported that dO_2_ concentrations below 10% were conducive to active P450 expression and Vail and co-workers reported that high dO_2_ concentrations led to an increase in misfolded protein compared with lower concentrations, and even used a concentration <1% for cultivation. Lu and co-workers found, however, that it was important not to limit dissolved oxygen levels [39,46,51].

The article "Recombinant production of eukaryotic cytochrome P450s in microbial cell factories" was published in 2018. Journal: Biosci Rep.

#### Conclusions on the production of eukaryotic P450s in *E. coli*

Table 2 summarizes the most successful strategies of recombinantly expressing P450s in *E. coli*, including expression systems and cultivation parameters used. The ten studies presented are the ones where product titers were especially high, a more comprehensive version of this table can be found in the Supplementary material. The tables focus on studies published in the past 20 years.

**Table 2:** Overview of strategies for P450 production in *E. coli*. Where plural strategies have been tested, the optimal one is marked in bold

P450	N-terminal modification	Coexpression	Volumetric titer	Yield	Reference
CYP4B1	**MALLLAVF**	–	660 nmol/l		[52]
CYP2E1	–	–	900–1400 nmol/l	14 nmol/mg protein	[53]
CYP154E1	–	Pdx/PdR and YkuN/FdR	825 nmol/l		[45]
CYP51F1	Truncation (2–37)	GroEL/GroES	1255 nmol/l		[24]
CYP61A1	Truncation (2–36)	GroEL/GroES	761 nmol/l		[24]
CYP505D6	–	GroEL/GroES	665 nmol/l		[24]
CYP505D8v1	–	GroEL/GroES	1333 nmol/l		[24]
CYP512E1	Truncation (2–8)	GroEL/GroES	973 nmol/l		[24]
CYP5137A4v1	–	GroEL/GroES	1820 nmol/l		[24]
CYP5139D7v1	Truncation (2–13)	GroEL/GroES	1230 nmol/l		[24]
CYP5147B1	Truncation (2–8)	GroEL/GroES	1310 nmol/l		[24]
CYP5150A2	Truncation (2–14)	GroEL/GroES	1020 nmol/l		[24]
CYP5037B3	NTD of CYP5144C1	GroEL/GroES	1213 ± 53 nmol/l		[24]
CYP5037E1v1	NTD of CYP5144C1	GroEL/GroES	2330 ± 44 nmol/l		[24]
CYP5146A1	NTD of CYP5144C1	GroEL/GroES	1041 ± 118 nmol/l		[24]
CYP5149A1	NTD of CYP5144C1	GroEL/GroES	2172 ± 62 nmol/l		[24]
CYP5037D1v1	NTD of CYP5144C1	GroEL/GroES	1213 nmol/l		[25]
CYP5037D1v2	NTD of CYP5144C1	GroEL/GroES	1440 nmol/l		[25]
CYP5037E1v2	NTD of CYP5144C1	GroEL/GroES	1645 nmol/l		[25]
CYP5147A4	NTD of CYP5144C1	GroEL/GroES	1552 nmol/l		[25]
CYP2B4	–	–	812 nmol/l	17 nmol/mg protein	[54]
CYP2B1	N-terminal truncation (3–21), positive charges substituted	–	800–1000 nmol/l	19 nmol/mg protein	[55]
CYP2C9	Truncation	CPR	800 nmol/l		[39]
CYP1A2	Truncation	CPR	1010 nmol/l		[39]
CYP2C3	N-terminal truncation (3–20)	–	800–1200 nmol/l	17 nmol/mg protein	[56]
CYP2W1	Various N-terminal modification, **rabbit P450 sequence (MAKKTSSKGK)**	GroEL/GroES	1800 nmol/l	16.8 nmol/mg protein	[48]

The highest volumetric titer reported was found by Ichinose and co-workers who achieved product yields of more than 2000 nmol/l when expressing the fungal P450s, CYP5037E1, and CYP5149A1, in *E. coli*. The P450s were N-terminally modified, creating a chimeric version with the N-terminal domain of CYP5144C1. Chaperones were coexpressed with the product and a membrane tolerant *E. coli* strain (C41(DE3)) was employed. However, the same strategy proved unsuccessful for other fungal P450s, including CYP5037B4 and CYP5037E5, where no expression was detected [24,25]. Ichinose et al. [25] also showed that with a similar strategy, only applying coexpression of chaperones and using *E. coli* strain C41(DE3), exceptionally high yields of 1820 nmol/l were achievable for CYP5137A4v1.

The article "Recombinant production of eukaryotic cytochrome P450s in microbial cell factories" was published in 2018. Journal: Biosci Rep.

High product yields were also found by Wu and co-workers who used a combination of expression strategies as well: the protein was N-terminally modified, by exchanging the native N-terminal region, before the proline rich hinge, with the N-terminal region of CYP2C3, which stems from rabbit, and had been used for successful soluble expression before. Aside from the N-terminal modification, this study also utilized the coexpression of the chaperones GroES/EL, which was shown to increase production from 350 to 1800 nmol/l. However, the same strategy was also applied to a second P450 (CYP2W1), where it only led to moderate levels of 600 nmol/l [48].

The membrane protein tolerant *E. coli* strain C41(DE3), used by Ichinose et al. [24,25], was also used by Cheng et al. [53] for expression of native CYP2E1, where it similarly led to exceptionally high product titers of 900–1400 nmol/l cell culture.

Concluding it seems that production of P450s in *E. coli* can be boosted most successfully by employing membrane protein tolerant strains and by coexpressing chaperones for elevated yields of active, correctly folded product. Aside from that, engineering a protein variant with an N-terminus of a P450, which has already been successfully expressed in soluble form, seems advantageous.

### Yeasts

Yeasts, especially *P. pastoris* and *S. cerevisiae*, are frequently used hosts for the recombinant expression of proteins. For both expression systems, fast and easy genetic manipulation tools are available. Yeast can be cultivated rather quickly up to high cell densities. In contrast to *E. coli*, yeasts are able to perform many post-translational modifications (although e.g. the glycosylation is different from humans or other eukaryotes) and they possess similar inner organelles as other eukaryotes, allowing proper anchoring of membrane bound proteins [57,58]. An overview of strategies for P450 expression is given in Figure 6.

**Figure 6:** Strategies for recombinant expression of P450s in yeasts Overview of strategies applied for the expression of P450s in yeasts.

#### N-terminal modifications

When expressing P450s in yeasts, as opposed to *E. coli*, the N-terminal anchor is less of an obstacle. Yeasts provide an environment more suitable for the expression of eukaryotic membrane bound proteins, as they are equipped with inner organelles, including the endoplasmic reticulum and mitochondria, where the proteins can anchor [58]. However, membrane space is limited, and thus production might still be enhanced and purification can be tremendously facilitated, when soluble variants of the proteins are engineered. This has, for instance, been done by Schoch and co-workers who engineered a soluble version of plant CYP73A1: the N-terminus was replaced by the peptitergent, amphipathic sequence PD1. This allowed simplification of purification, improved solubility and stability in the absence of detergents, and allowed structure investigations by NMR [59].

The article "Recombinant production of eukaryotic cytochrome P450s in microbial cell factories" was published in 2018. Journal: Biosci Rep.

#### Coexpression of CPR and other proteins

Yeasts, in contrast to *E. coli*, do natively inhere CPRs. However, overexpression of P450s entails a disproportionately high demand for NADP. Therefore, co-overexpression of CPRs is a frequently used strategy. For instance, Chandor-Proust and co-workers engineered a strain simultaneously expressing mosquito CYP6Z8 and cytochrome P450 reductase, and achieved a titer of 17 mg/l [60].

In some cases, previously engineered *S. cerevisiae* strains, which already overproduced CPRs, were used. For instance, Ducassou and co-workers compared three strains, one overexpressing yeast CPR (W(R)), one overexpressing human CPR (W(hR)), and one expressing yeast CPR (W(N)), and found the highest amount of active human P450 2U1 in the strain overexpressing human cytochrome reductase besides the P450 [61]. In contrast, Stegemann et al. [62] used the *Saccharomyces* strain W(R), which overexpresses yeast cytochrome reductase, for enhanced expression of 5 P450s from Zebrafish. Hamann et al. [63] used an engineered *S. cerevisiae* strain WAT11, which expressed the *Arabidopsis thaliana* CPR, for successful expression of two plant P450s. Truan and co-workers coexpressed mammalian P450s together with varying amounts of CPRs and cytochrome *b*_5_ and found that the activity of all P450s increased with higher amounts of CPR present. For some P450s also the coexpression of cytochrome *b*_5_ was beneficial [64].

With the ultimate goal of substrate conversions, coexpression of P450 and CPR can be beneficial, as deprivation of a redoxpartner is unlikely. Garrait et al. [65] engineered a *S. cerevisiae* strain, for coexpression of plant P450 73A1 and CPR, which allowed conversion of cinnamic acid to coumaric acid. Nazir et al. [66] constructed a library of 121 isoforms of cytochrome P450 monooxygenases from *Aspergillus oryzae*, and coexpressed them together with NADPH-cytochrome reductase in *S. cerevisiae* to find new catalytic functions. Syed et al. [67] were able to identify six fungal P450 monooxygenases that oxidize polycyclic aromatic hydrocarbons when simultaneously expressing the P450s together with CPR in *P. pastoris*.

The article "Recombinant production of eukaryotic cytochrome P450s in microbial cell factories" was published in 2018. Journal: Biosci Rep.

The production of ortho-hydroxydaidzein derivatives was achieved by Chang and co-workers, when fusing the reductase domain of the bacterial CYP102A1 to the fungal CYP57B3, and expressing the fusion protein actively in *P. pastoris* [68].

#### Conclusions on the production of eukaryotic P450s in yeasts

Table 3 summarizes P450 expression-studies in yeast. Per species three studies with exceptionally high product yields are presented. A more comprehensive version of this table can be found in the Supplementary material. The tables focus on studies published in the past 20 years.

**Table 3:** Overview of strategies for P450 production in *S. cerevisiae* and *P. pastoris*. Where two or more strategies have been tested, the optimal one is marked in bold

P450	N-terminal modification	Coexpression	Yield	Reference
***S. cerevisiae***				
CYP79A1	Optimized 14 codons at 5′ end	CPR	50–330 pmol/mg protein	[63]
CYP71E1	Optimized 13 codons at 5′ end	CPR	50–330 pmol/mg protein	[63]
CYP71D18	Tried N-terminal modifications but less expressed than with native construct	CPR	400 pmol/mg protein	[14]
CYP73A1	**PD1-sequence**	CPR	369 pmol/mg protein	[59]
***P. pastoris***				
CYP2D6	–	CPR	0.12 nmol/mg protein	[69]
CYP5136A2	–	CPR	75–275 pmol/ mg protein	[67]
CYP5145A3	–	CPR	75–275 pmol/ mg protein	[67]
CYP5144A7	–	CPR	75–275 pmol/ mg protein	[67]
CYP5136A3	–	CPR	75–275 pmol/ mg protein	[67]
CYP5142A3	–	CPR	75–275 pmol/ mg protein	[67]
CYP5144A5	–	CPR	75–275 pmol/ mg protein	[67]
CYP17	–	–	300 pmol/ mg microsomal protein	[70]

In general, higher P450 yields have been achieved in *S. cerevisiae*, compared with the studies conducted in *P. pastoris*. In almost all studies presented in Table 3, CPR was co-overexpressed. N-terminal modifications seem to have varying impacts on upstream processing, while their main impact definitely applies to downstream processing, which is facilitated tremendously if the target protein is not anchored in the membrane.

### *E. coli* verses yeasts

To date, many more studies have been conducted using *E. coli* as expression systems compared to yeasts. This might be explicable, as *E. coli* is easier to cultivate and grows much faster than yeasts. Also more tools for genetic manipulation are available, and procedures are less time-consuming and laborious. However, when having a look at the features of eukaryotic P450s in particular, it is still surprising that *E. coli* has been chosen over yeasts. Most eukaryotic P450s natively carry a membrane anchor, making protein engineering almost inevitable when expressing the proteins in *E. coli*. Yeasts, on the other hand, provide the necessary environment for anchoring membrane proteins, which makes active expression of the P450 more straightforward. Nevertheless, when expressing the P450 including its native N-terminal region, downstream processing is not as effortless as the membrane has to be solubilized. Thus, protein engineering might not be easily circumvented either way.

The article "Recombinant production of eukaryotic cytochrome P450s in microbial cell factories" was published in 2018. Journal: Biosci Rep.

A direct comparison of heterologous hosts for P450 expression has been conducted by Haudenschild and co-workers who compared expression of three different P450s from mint in *S. cerevisiae* and *E. coli.* They found the results summarized in Table 4. The data presented for expression in *E. coli* results from P450s that were N-terminally modified (five residues were N-terminally deleted and replaced with nine residues from the MALLLAVFL-sequence), while in *S. cerevisiae* the native P450s were expressed. For CYP71D18 also expression of the native construct in *E. coli* was tested. However, no P450 could be detected by CO-difference spectrometry [14].

**Table 4:** Comparison of the expression of P450 from mint in *E. coli* and *S. cerevisiae* [14]

P450	*E. coli*		*S. cerevisiae*	
	Titer (nmol/l)	Yield (pmol/mg protein)	Titer (nmol/l)	Yield (pmol/mg protein)
CYP71D18	350	810	n.d.	527
CYP71D15	500	1400	0	50
CYP71D13	265	420	14	66

As shown in Table 4, for two out of the three P450s investigated, expression in *E. coli* led to much higher yields. The same trend is deducible from Tables 2 and 3, which show that the highest yields reached in *E. coli* lie in the range of 14–20 nmol/mg protein [48,53–56] while the highest yields in yeast are all below 1 nmol/mg protein [14,59,63,67,69,70]. However, those yields are hard to compare as the P450 expressed in yeasts are all expressed in their native form, while the majority of the ones expressed in *E. coli* are N-terminally modified.

## Conclusions

Up to now, many strategies have been developed for the expression of active P450s in microbial cell factories that enhance the yields of active protein. However, the success of such strategies seems to depend on each single P450 to be expressed. Some sequences, such as the MALLLAVF-sequence, have proven effective in several cases, e.g. [11–15]. For example, changing the N-terminal region to this sequence helped increasing the titer of CYP6G1 from 0 nmol/l (native construct) to 460 nmol/l [13] or in case of CYP71D18 from 0 nmol/l (native construct) to 350 nmol/l [14]. However, application of this strategy did not always lead to the highest product yields [21–23,50]. For instance Gillam et al. [22] achieved a more than 20-fold higher yield when performing deletions in the N-terminal region of CYP2E1, compared with using the bovine sequence. Also when it comes to coexpression of CPRs, varying results were observed. In many cases the coexpression of CPRs led to formation of high titers of active P450 [12,29,39] (up to 1010 nmol/l). However, in other cases the product titer was clearly decreased (more than 4-fold, from 460 to 97 nmol/l) when coexpressing the redoxpartner [13].

The article "Recombinant production of eukaryotic cytochrome P450s in microbial cell factories" was published in 2018. Journal: Biosci Rep.

To sum this up, there are several strategies available to achieve high-level expression, which have already been shown for certain P450s; however, for the expression of a novel P450 protein, different strategies might have to be applied for an optimal outcome. In *E. coli* the most promising strategies include using a membrane-protein tolerant strain (C41(DE3)), and coexpressing chaperones for correct folding of the P450. Also, exchanging the N-terminal domain for that of an existing soluble P450 is a promising strategy for obtaining active protein. To date, highest P450 yields in *E. coli* lie in the range of 14 to19 nmol/mg protein [48,53–56]. In yeasts, most successful approaches involve the co-overexpression of cytochrome reductase. N-terminal modifications mainly seem to have an impact on facilitated purification. In those heterologous hosts, highest P450 yields currently lie between 75 and 400 pmol/mg protein [14,59,63,67,69,70]. In general, we believe that the means of bioprocess engineering, namely adjusting cultivation and induction conditions, represent a yet rather untapped potential for boosting the recombinant production of active P450s in the different hosts.

## Abbreviations

δ-ALA: δ-Aminolevulinic acid
CPR: cytochrome P450 reductase
IPTG: isopropyl-β-D-thiogalactopyranosid
P450: cytochrome P450
